The article "Comprehensive N-glycan profiles of hepatocellular carcinoma reveal association of fucosylation with tumor progression and regulation of FUT8 by microRNAs" was retracted in 2025. Reason: duplicated images.

# Comprehensive N-glycan profiles of hepatocellular carcinoma reveal association of fucosylation with tumor progression and regulation of FUT8 by microRNAs

**DOI:** 10.18632/oncotarget.11284

**Published:** 2016-08-13

**Authors:** Lei Cheng, Shuhang Gao, Xiaobo Song, Weijie Dong, Huimin Zhou, Lifen Zhao, Li Jia

**Affiliations:** ^1^ College of Laboratory Medicine, Dalian Medical University, Dalian 116044, Liaoning Province, China; ^2^ Department of Laparoscopic Surgery, The First Affiliated Hospital of Dalian Medical University, Dalian 116011, Liaoning Province, China; ^3^ Department of Oncology, The First Affiliated Hospital of Dalian Medical University, Dalian 116011, Liaoning Province, China; ^4^ Department of Medical Biology, Faculty of Health Sciences, University of Tromsø, Tromsø, Norway; ^5^ Department of Biochemistry, Dalian Medical University, Dalian 116044, Liaoning Province, China; ^6^ Department of Microbiology, Dalian Medical University, Dalian 116044, Liaoning Province, China

**Keywords:** fucosyltransferase (FUT) gene, human hepatocellular carcinoma cell lines, tumor progression, microRNAs

## Abstract

Glycosylation has significant effects on cancer progression. Fucosylation is one of the most important glycosylation events involved in hepatocellular carcinoma (HCC). Here, we compared N-glycan profiles of liver tumor tissues and adjacent tissues of 27 HCC patients to reveal the association between fucosylation and HCC progression, as well as verified the potential role of miRNA in regulating fucosylation. Mass spectrometry (MS) analysis showed pronounced differences of the N-glycosylation patterns and fucosylated N-glycans between the adjacent and tumor tissues. Different fucosyltransferase (FUT) genes were also identified in adjacent and tumor tissues, and two HCC cell lines with different metastatic potential. High-level expression of FUT8 was detected in tumor tissues and highly metastatic HCC cells. Altered levels of FUT8 in HCC cell lines significantly linked to the malignant behaviors of proliferation and invasion *in vitro*. Furthermore, using microRNA array, we identified FUT8 as one of the miR-26a, miR-34a and miR-146a-targeted genes. An inverse correlation was revealed between the expression levels of FUT8 and these miRNAs. Luciferase reporter assay demonstrated these miRNAs specifically interacted with the 3′UTR of FUT8 and subsequently down-regulated FUT8 expression-level. The forced expression of these miRNAs was able to induce a decrease in FUT8 levels and thereby to suppress HCC cells progression. Altogether, our results indicate that fucosylated *N*-glycan and FUT8 levels can be used as markers for evaluating HCC progression, as well as miRNAs may be involved in inhibition of fucosylation machinery through targeting FUT8.

## INTRODUCTION

Liver cancer is the 5th most common cancer, but the 2nd leading cause of cancer death. Approximately 80% of all liver cancers are hepatocellular carcinoma (HCC), which has very high mortality due to its poor early diagnosis and limited treatment. [1] Despite recent advances in disease management and treatment, the prognosis in HCC patients remains unfavorable with a median survival of most patients of 6–9 months after diagnosis [2]. Therefore, it is urgent to investigate the molecular mechanism of HCC so as to identify markers for HCC diagnosis and targets for effective therapeutic strategies.

Glycosylation is a common and highly diverse form of protein modification [3]. Altered glycosylation is a hallmark of cancer that is found to occur during cancer progression [4, 5]. Glycans are detected in many cancer-associated events such as migration, adhesion, and metastasis [6]. Aberrant glycosylation and increased fucosylation are lately recognized as an indicator of HCC. Zhang *et al.* showed that the fucosylated glycans were upregulated in HCC serum samples versus cirrhosis samples [7], and the level of core-α-1, 6-fucosylated glycan increased both on the cell surface and in the serum samples of HCC patients [8]. Mehta *et al.* found that the N-linked glycans varied when comparing 16 tumor samples and adjacent tissue of HCC [9]. Zhu *et al.* demonstrated that aberrant fucosylation of glycosphingolipids in HCC overexpressed in tumor tissues in comparison to peritumoural tissues [10]. Investigation of HCC-associated glycosylation changes can be vital for better understanding of the function of fucosylated glycans and fucosyltransferases (FUTs) in the progression of HCC.

FUT family is a group of fucosylation synthases. So far, 13 FUTs are known to be encoded in the human genome, i.e. FUT1 to 11, protein O-FUT 1 (POFUT1), and POFUT2 [11]. Forced FUT1 expression in human hepatocarcinoma cells led to the inhibition of tumor growth [12], and FUT2 expression was found increased in HCC cells [13]. FUT6 was highly expressed in HCC tissues and positively associated with the progression of HCC cells [14]. FUT7 was a potential anti-apoptotic factor in human hepatocarcinoma cells [15]. FUT8 was also up-regulated in HCC, and associated to hepatocarcinogensis and poor differentiation [16, 17]. Although FUT family is well-known to play an important role in HCC progression, the underlying mechanisms of fucosylation mediated by miRNA remain unknown.

MicroRNAs (miRNAs) are evolutionarily conserved noncoding RNAs of 21–25 nucleotides in length, with function as critical gene regulators via negatively regulating the expression of target genes [18]. Recent studies have identified several deregulated miRNAs in HCC tissues or cells, and revealed their activities in HCC carcinogenesis and progression. Altogether indicates that restoration of the deregulated miRNAs might be considerable therapeutic strategies for HCC [19, 20]. Among the HCC-related miRNAs, contradictory relationship between miR-34a or miR-26a levels and HCC malignance was reported. MiR-34a expression was significantly decreased in HCC compared with those in corresponding adjacent tissues, and it was found associated with malignant characteristics in patients with HCC [21, 22]. The miR-26a expression was significantly down-regulated in HCC cells and HCC tissues, and overexpression of miR-26a promoted apoptosis of HCC cells [23, 24]. However, it is unclear whether miR-34a, miR-26a and miR-455-3p can inhibit the malignant behaviors of HCC cells through fucosylation mediation.

Here, we obtained the comprehensive *N-*glycan profiles and fucosylated *N*-glycan alteration of adjacent and tumor tissues from HCC patients using MALDI-TOF-MS analysis. Expression level of FUT genes was measured between the tumor samples and adjacent tissues, and HCC cells with different metastatic potential using real-time PCR. In addition, miR-26a, miR-34a and miR-146a-targeted genes were identified with microRNA array. This study provides new insights into HCC-associated fucosylated *N*-glycan changes and sets a miRNA-mediated mechanism.

## RESULTS

### Comparison with *N*-glycans derived from HCC tumor and adjacent tissues

In this study, 27 HCC tumor tissues and corresponding adjacent tissues were applied to study the HCC-specific, cell-surface N-glycans by using MALDI-TOF MS analysis. *N-*glycan profile spectra of HCC tumor and adjacent tissues were shown in Figure 1A. The assigned *N*-glycan signals were summarized in Table 1. The intensities of the observed MS signals were presented as a histogram in Figure 1B labeled with the estimated monosaccharide composition. The results showed that the *N*-glycan profiles of HCC tissues were substantially distinguished from those of the corresponding adjacent tissues (Figure 1A). The *N-*glycan profiles of HCC tumor and adjacent tissues were dominated by high-mannose type glycans (peak 4, 8, 12, 15 and 17, Table 1). The ten most abundant *N*-glycans peak 1, 5, 9, 10, 14, 16, 20, 21, 24 and 25 were identified exclusively in tumor tissues (Table 1), amongst peak 1, 5, 9, 16, 20, 21, 24 and 25 were of fucosylated *N*-glycans. Peak 18 was also significantly increased in the tumor group (> 2 fold) compared to the adjacent tissue group (Figure 2B). The levels of peaks 6, 7, 12, 15, 17, 19, 22, and 23 were significantly increased in the adjacent tissue group (> 2 fold) compared to the tumor group (Figure 2B), but only peak 22 was shown to be fucosylated *N*-glycans. Notably, the peaks corresponding to fucosylated oligosaccharides were often observed in tumor tissues.

**Figure 1:** The profiles of *N*-Glycan composition in HCC tumor and adjacent tissues (**A**) MALDI-TOF MS spectra of *N*-glycans from HCC tumor and adjacent tissues were shown respectively. *N*-glycans were released by PNGase F and permethylated. (**B**) Histograms of relative intensities of the differential *N*-glycan signals were observed (the histograms represents only signal intensities but not the quantities). The signals indicated with Arabic numerals are summarized in Table 1.

**Table 1:** N-glycans analyzed in tumor and adjacent tissues by MALDI-TOF MS

Glycan number	Observed m/z		Chemical composition
	adjacent	tumor	
1	No	1345.712	Fuc+Man_3_HexNAc_2_
2	1375.708	1375.723	Hex+Man_3_HexNAc_2_
3	1416.727	1416.754	HexNAc+Man_3_HexNAc_2_
4	1579.797	1579.831	Man_2_+Man_3_HexNAc_2_
5	No	1590.847	HexNAcFuc+Man_3_HexNAc_2_
6	1620.824	1620.846	HexHexNAc+Man_3_HexNAc_2_
7	1661.848	1661.886	HexNAc_2_+Man3HexNAc_2_
8	1783.901	1783.936	Man_3_+Man_3_HexNAc_2_
9	No	1794.958	HexHexNAcFuc+Man_3_HexNAc_2_
10	No	1824.957	Hex_2_HexNAc+Man_3_HexNAc_2_
11	1835.969	1835.985	HexNAc_2_Fuc+Man_3_HexNAc_2_
12	1988.007	1988.039	Man_4_+Man_3_HexNAc_2_
13	2010.003	2010.062	HexNAc2Fuc2+Man3HexNAc2
14	No	2070.094	Hex_2_HexNAc_2_+Man_3_HexNAc_2_
15	2192.110	2192.152	Man_5_+Man_3_HexNAc_2_
16	No	2244.198	Hex_2_HexNAc_2_Fuc+Man_3_HexNAc_2_
17	2396.206	2396.254	Man_6_+Man_3_HexNAc_2_
18	2407.173	2407.231	Hex_4_HexNAcFuc+Man_3_HexNAc_2_
19	2431.223	2431.284	Hex_2_HexNAc_2_NeuAc+Man_3_HexNAc_2_
20	No	2605.378	Hex_2_HexNAc_2_FucNeuAc+Man_3_HexNAc_2_
21	No	2693.424	Hex_3_HexNAc_3_Fuc+Man_3_HexNAc_2_
22	2768.339	2768.398	Hex_4_HexNAcFucNeuAc+Man_3_HexNAc_2_
23	2792.423	2792.448	Hex_2_HexNAc_2_NeuAc_2_+Man_3_HexNAc_2_
24	No	2966.557	Hex_2_HexNAc_2_FucNeuAc_2_+Man_3_HexNAc_2_
25	No	3054.615	Hex_3_HexNAc_3_FucNeuAc+Man_3_HexNAc_2_

**Figure 2:** Differential expression of FUT family in HCC tissues and HCC cell lines The mRNA levels of FUT family were analyzed by qRT-PCR. (**A**) Tumor tissues expressed higher levels of FUT4, FUT5, FUT8, FUT11 and POFUT2 mRNA than adjacent tissues. (**B)** MHCC97H cells with high metastatic potential expressed higher levels of FUT4, FUT5, FUT6 and FUT8 mRNA than MHCC97L cells with low metastatic potential. Data are the means ± SD of triplicate determinants.

### Differential expression of FUT family in HCC tissues and HCC cell lines

To increase our understanding of the regulation of fucosylation, the mRNA levels of FUT family were obtained by qRT-PCR in the HCC tumor and adjacent tissues. Our data demonstrated that tumor tissues contained higher levels of FUT4 (2.19 folds), FUT5 (1.81 folds), FUT8 (2.76 folds), FUT11 (2.03 folds) and POFUT2 (1.55 folds) transcripts compared to adjacent tissues (Figure 2A). No significant difference was shown in the expression level of the other members of FUT family between the two groups except FUT1 (1.64 folds), FUT2 (1.58 folds) and FUT7 (1.75 folds) high in the adjacent tissues (Figure 2A).

Furthermore the FUT family was examined in two HCC cell lines. The FUT gene expression levels of the MHCC97H cells with high metastatic potential differed from cell lines MHCC97L with low metastatic potential. MHCC97H cells showed a remarkable increase in mRNA level of gene FUT4 (2.84 folds), FUT5 (2.03 folds), FUT6 (1.67 folds), and FUT8 (3.11 folds) (Figure 2B), suggesting that MHCC97H cells expressed high levels of fucosylation-related genes. Only slight difference was observed in the level of FUT1 (1.75 folds) and FUT9 (1.58 folds) mRNA. No significant differences were found in the transcription level of FUT2, FUT3, FUT7, FUT10, FUT11, POFUT1 and POFUT2 mRNA (Figure 2B). In the current study FUT8 of 3.11 folds expression was chosen for further investigation.

### FUT8 correlates with HCC cells progression

In order to understand whether FUT8 has biological significance in the progression of HCC cells, highly metastatic MHCC97H cells were subjected to FUT8 knockdown, while low metastatic MHCC97L cells were stably transfected with FUT8. Both were examined for tumor progression *in vitro*. As shown in Figure 3A, the expression of FUT8 was significantly decreased both in transcription and protein level in MHCC97H shFUT8 transfectant compared with those in the controls. The higher expression levels of FUT8 were detected in MHCC97L FUT8 cells (Figure 3C).

**Figure 3:** FUT8 correlates with HCC cells progression *in vitro* (**A**) FUT8 transcript was decreased apparently in MHCC97H cells by shRNA treatment. The distinct reduction of FUT8 was observed at mRNA and protein levels by qRT-PCR and western blot analysis (*P < 0.05). (**B**) Differential FITC-LCA binding profiles of MHCC97H control and MHCC97H shFUT8 cell lines using flow cytometry. Histograms of fluorescence intensities of cells with specific carbohydrate expression as determined. (**C**) After full-length sequences transfection, FUT8 mRNA and protein levels were increased notably in MHCC97L cells by qRT-PCR and western blot analysis (*P < 0.05). (**D**) Flow cytometry analysis showed α-1, 6 fucosylation level detected by FITC-LCA on the cell surface, was also increased in MHCC97L FUT8 cells. (**E**) Growth curves of MHCC97H shFUT8 cells were compared to control cells with the CCK-8 assay. (**F**) Transwell cell migration and invasion assays were performed to compare cell migration and invasion between MHCC97H shFUT8 cells and MHCC97H control. (**G**) Growth curves of MHCC97L FUT8 cells were compared to control cells with the CCK-8 assay. (**H**) *In vitro* Transwell cell migration and invasion analysis was performed. MHCC97L FUT8 cells were significantly more migratory and invasive (*P < 0.05) than MHCC97L mock cells. Data are the means ± SD of triplicate determinants (*P < 0.05).

LCA lectin, which recognizes Fucα-1, 6GlcNAc structures (product of FUT8), was used to analyze the alterations in the *N*-glycosylation pattern of glycoproteins. We examined the fluorescence intensity of FITC-LCA-lectin binding on MHCC97H and MHCC97L cells after FUT8 regulation using flow cytometry. Figure 3B showed that the FUT8 knockdown resulted in a decrease of α-1, 6 fucosylation level in MHCC97H shFUT8 cells. The fluorescence intensity on FITC-LCA also revealed variation of α-1, 6 fucosylation in MHCC97L FUT8 cells compared with those in the controls (Figure 3D).

As expected, cell counting kit-8 (CCK-8) assays revealed that knockdown of FUT8 repressed MHCC97H shFUT8 proliferation (Figure 3E). Inversely, overexpression of FUT8 promoted MHCC97L FUT8 cells proliferation (Figure 3G). We next assessed the effect of FUT8 on cell migration and invasion. Down-regulation of FUT8 using shRNA resulted in a significant decrease in the migratory and invasive capabilities of MHCC97H shFUT8 cells (Figure 3F), and overexpressing FUT8 in MHCC97L resulted in a significant increase in the percentage of migratory and invasive cells (Figure 3H). Overall our results demonstrated that FUT8 indeed mediated tumor cells progression *in vitro* through modifying the N-glycosylation profile in terms of Fucα-1, 6GlcNAc structures in HCC cells.

### MiR-26a, miR-34a and miR-455-3p directly target FUT8

Recent studies have linked tumor progression to the altered expression of miRNAs. We first screened the expression profiles of human miRNAs in MHCC97H and MHCC97L cell lines using microRNA array (Kangchen, Shanghai, China). The studies indicated that 3 microRNAs (miR-26a, miR-34a, and miR-455-3p) were down-regulated by at least 2 fold in the MHCC97H cells compared to those in the MHCC97L cells. To explore and confirm the findings from our microRNA array analysis, we examined the expression levels of miRNAs in HCC cell lines and HCC samples by qRT-PCR. The results in Figure 4A show remarkably lower levels of miR-26a, miR-34a, and miR-455-3p in 27 HCC tissues than in adjacent tissues. These miRNAs were also underexpressed in MHCC97H cells compared to those in MHCC97L cells and L02 cells (Figure 4B). This suggested that down-regulation of miR-26a, miR-34a, and miR-455-3p might be involved in the progression of HCC. We then examined the relationship between miR-26a, miR-34a, miR-455-3p and FUT8 expression in 27 HCC tissue samples by qRT-PCR. As shown in Figure 4C, the FUT8 mRNA expression appeared to be inversely correlated with the levels of miRNAs (*P* < 0.05), which was consistent with HCC cell lines. FUT8 mRNA was also overexpressed in 27 HCC tissues compared to adjacent tissues (Figure 4D).

**Figure 4:** MiR-26a, miR-34a and miR-455-3p as negative regulators of FUT8 (**A**) miR-26a, miR-34a and miR-455-3p expression were significantly decreased in 27 HCC compared with the corresponding adjacent tissues using qRT-PCR analysis. (**B**) The expression of miR-26a, miR-34a and miR-455-3p was examined by qRT-PCR in the MHCC97H, MHCC97L and L02 cell lines. (**C**) Relationship between miR-26a, miR-34a and miR-455-3p levels and FUT8 mRNA expression in 27 HCC tumor and 27 adjacent tissues. (**D**) FUT8 expression was significantly increased in 27 HCC compared with the corresponding adjacent tissues using qRT-PCR analysis. (**E**–**G)**. The nucleotides sequence of the target site of miRNAs in FUT8 3′-UTR was shown; Luciferase assay for the direct targeting of 3′-UTR of FUT8 by miR-26a, miR-34a and miR-455-3p. The wide-type and mutant miRNA target sequences of FUT8 were fused with luciferase reporter and transfected into 293T cells, transfected with miRNA mimic and NC mimic. The mean of the results from the cells transfected with the NC mimic was set at 100. Each bar represents the relative luciferase activity (*P < 0.05). (**H**) FUT8 was analyzed by qRT-PCR and western blot in MHCC97H cells treated with miR-26a, miR-34a and miR-455-3p mimic (*P < 0.05). (**I**) FUT8 was analyzed by qRT-PCR and western blot in MHCC97L cells treated with miR-26a, miR-34a and miR-455-3p inhibitor (*P < 0.05). Data are the means ± SD of triplicate determinants.

Next, we investigated whether the 3′UTR of FUT8 is a direct target of miR-26a, miR-34a, and miR-455-3p. To do so, the complementary sequence to miR-26a, miR-34a, or miR-455-3p seed sequence of FUT8 3′-UTR (wt 3′-UTR) was cloned into a luciferase reporter vector. In parallel, we mutated the 3′UTR of FUT8 (mut 3′-UTR) complementary to the miR-26a, miR-34a, or miR-455-3p seed sequence in the same reporter plasmid. HEK-293 cells were then transfected with wt or mut FUT8-3′UTR vector and miR-26a, miR-34a, or miR-455-3p mimics. Forced miRNAs expression decreased luciferase activity, and this suppression was reversed by the mutation of the target sequences in the 3′-UTRs of FUT8 (Figure 4E–4G).

We further transfected MHCC97H cells with miR-26a, miR-34a, or miR-455-3p mimics, MHCC97L cells with inhibitor and measured the changes in FUT8 expression levels. Overexpression of miR-26a, miR-34a, or miR-455-3p remarkably reduced FUT8 expression both mRNA and protein levels in MHCC97H cells (Figure 4H). Conversely, knockdown of miR-26a, miR-34a, or miR-455-3p increased the expression level of FUT8 in MHCC97L cells (Figure 4I). Taken together, these results suggest that miR-26a, miR-34a, and miR-455-3p directly bind and negatively regulate FUT8 mRNA stability.

### MiR-26a, miR-34a and miR-455-3p regulate HCC progression by targeting FUT8

Since miR-26a, miR-34a and miR-455-3p targeted FUT8, we further investigated whether these miRNAs modulated HCC progression and the underlying mechanisms. As shown in Figure 5A, mimics of these miRNAs strongly up-regulated miR-26a, miR-34a and miR-455-3p expression in MHCC97H cells. The effect of miRNAs overexpression markedly inhibited MHCC97H cells proliferation and colony formation efficiency (Figure 5B, 5C). Because Ki67 antigen is an important marker of cell proliferation, we next examined Ki67 expression by immunofluorescence analysis. The staining results showed that the overexpression of miRNAs in MHCC97H cells significantly down regulated Ki67 staining (Figure 5D). We next assessed the effects of miRNA on MHCC97H cell migration and invasion. Overexpression of miR-26a, miR-34a and miR-455-3p significantly decreased the migration and invasion abilities of MHCC97H cells (Figure 5E).

**Figure 5:** Effect of miR-26a, miR-34a and miR-455-3p mimic on cell progression in MHCC97H cells (**A**) The expression of miR-26a, miR-34a and miR-455-3p was studied by qRT–PCR in MHCC97H cells transfected with the mimics (*P < 0.05). (**B**) Transfection of miR-26a, miR-34a and miR-455-3p mimic in MHCC97H cells inhibited cellular viability as revealed by CCK-8 assay (*P < 0.05). (**C**) Overexpression of miR-26a, miR-34a and miR-455-3p inhibited the growth of MHCC97H cells with in focus formation assay. (**D**) Ki67 expression was detected by immunofluorescence staining in MHCC97H cells treated with miRNA mimic transfection. Red fluorescence: Ki67; DAPI staining for nuclear DNA. (**E**) Transwell cell migration and invasion assays were used to compare cell migration and invasion between miRNA mimic- and NC mimic-transfected cells. The data were mean ± S.D. of three separate transfections (*P < 0.05).

Anti-miRNAs were transfected into MHCC97L cells followed by qRT-PCR and western blot analysis. As shown in Figure 6A, inhibitor of these miRNAs decreased the expression of miR-26a, miR-34a and miR-455-3p in MHCC97L cells. CCK-8 assays revealed that MHCC97L cells in the miRNA inhibitor groups had higher proliferative ability than controls (Figure 6B). The colony formation and Ki67 expression were also increased in the miRNA inhibitor groups (Figure 6C, 6D). Matrigel invasion and migration assays were also performed, and exogenously downregulation of miRNA expression increased the number of invasive and migratory cells significantly (Figure 6E).

**Figure 6:** Effect of miR-26a, miR-34a and miR-455-3p inhibitor on cell progression in MHCC97L cells (**A**) The expression of miR-26a, miR-34a and miR-455-3p was studied by qRT–PCR in MHCC97L cells transfected with the inhibitor (*P < 0.05). (**B**) MHCC97L cells were transfected with miR-26a, miR-34a and miR-455-3p respectively. Expression of miRNA was confirmed by qRT–PCR. B, Growth curves of miRNA inhibitor-transfected cells were compared to NC inhibitor cells with the CCK-8 assay (*P < 0.05). (**C**) Morphology foci were observed at the microscope and photographed. (**D**) Ki67 expression was detected by immunofluorescence staining in MHCC97L cells treated with miRNA inhibitor transfection. Red fluorescence: Ki67; DAPI staining for nuclear DNA. (**E**) Knockdown of miR-26a, miR-34a and miR-455-3p significantly increased the migration and invasion of MHCC97L cells. The data were mean ± S.D. of three separate transfections (*P < 0.05).

To further determine whether miRNAs regulated MHCC97H cells tumorigenesis by targeting FUT8, we assessed the effects of miRNA mimics on MHCC97H cells xenograft formation. MHCC97H cells were transfected with miRNA mimics or NC mimic and implanted subcutaneously into the right flank of each nude mouse respectively (*n* = 6). One week later, the mice were intratumorally injected with mimic control or miR mimic three times per week for three weeks. Tumor sizes were measured with weekly after implantation. The result showed significantly reduced tumor volume and weight in miR-26a, miR-34a or miR-455-3p mimic expressing xenografts as compared to controls (*p* < 0.05) (Figure 7A). Consistent with the *in vitro* assay, we demonstrated that miR-26a, miR-34a and miR-455-3p significantly reduced the protein levels of FUT8 and Ki67 in the tumor tissues (Figure 7B).

**Figure 7:** MiR-26a, miR-34a and miR-455-3p mediates MHCC97H cells tumorigenesis by targeting FUT8 (**A**) MHCC97H cells were transfected with miRNA mimics or NC mimic and implanted subcutaneously into the right flank of each nude mouse respectively (*n* = 6). One week later, the mouse in groups were injected intratumorally with miRNA mimics or NC mimic three times per week for 3 weeks respectively. miR-26a, miR-34a and miR-455-3p inhibited the tumorigenesis of MHCC97H cells *in vivo*. The tumor volumes and weight were reduced in miRNA mimic groups to compare with NC mimic group (*P < 0.05). (**B**) The expression levels of Ki67 and FUT8 were analyzed by IHC in tumors.

## DISCUSSION

Representing the third class of biomacromolecules, glycans are becoming increasingly important in biological, chemical and clinical research and applications. Enhanced fucosylation has been proposed as a marker of the progression from liver disease to HCC. In the current study, we analyzed the characteristic *N*-linked profiling pattern and fucosylated *N*-glycan in HCC tissue samples. We further examined expression of FUT family, which was reported to be associated with tumor progression. We also showed that negative regulators of FUT8, such as miR-26a, miR-34a and miR-455-3p, could reduce FUT8-mediated progression in HCC.

Altered expression of *N*-glycans has been observed by MS in many types of tumor cells. MS technology as a novel methodology provides highly sensitive and rapid glycan analysis. *Holst* et al. have shown noticeable differences between the *N-*glycosylation patterns of 25 different colorectal cancer cell lines, as well as between the patterns of colorectal tumor tissues and corresponding control tissues from 13 colorectal cancer patients by MALDI-TOF (/TOF)-MS analysis [25, 26]. Recent studies quantitatively profiled *N*-linked glycans from human serum of healthy controls and ovarian cancer patients by MALDI-TOF/MS and provided critical information on tumor biomarkers for screening of ovarian cancer [27]. In an effort to identify the altered patterns, we applied MALDI-TOF-MS to profile total *N*-glycans in HCC tissues and adjacent tissues, and found dramatic differences in *N*-glycans between these two groups. This result corresponded with our findings of differential *N*-glycan composition in human HCC cell lines MHCC97H and MHCC97L with different metastatic potential by MS analysis [28]. Furthermore, MALDI-TOF-MS analysis of *N*-glycan profiles demonstrated increased fucosylated *N*-glycan in HCC tissues. Other researchers have also observed increased levels of core and outer-arm fucose residues in the serum of patients with HCC [29] and HCC tissues [30]. Overall, observation of the tendency toward enhanced fucosylation would be important in the monitoring of tumor progression.

Increasing studies demonstrate that the alterations of fucosylation and the levels of fucosyltransferases activities derived from the malignant transformation are relevant to tumor progression and metastasis [31–34]. In the present study, the results indicated that the FUT profiling patterns were significantly different in HCC tissues to adjacent tissues. Among these the expression of FUT4, FUT5, FUT8, FUT11 and POFUT2 was significantly up-regulated in HCC tissues compared to adjacent tissues, and FUT8 was the most expressed on HCC tissues. As shown in recent research, the FUT8 mRNA level was significant higher in 24 pairs of HCC tissues than that in their corresponding adjacent non-tumor liver tissues [35]. In addition, the expression profiles of FUT gene family were shown to be remodeled in HCC cell lines. MHCC97H cell with high metastatic potential was characterized of higher levels of FUT4, FUT5, FUT6 and FUT8, while MHCC97L cell with low metastatic potential expressed more FUT1 and FUT9. FUT8 level was also found to be up-regulated in high metastatic potential HCCLM3 cells (HCC cell lines) in comparison to Hep3B cells [36]. Our results showed a significant correlation between N-glycan traits derived from MS-data and corresponding FUT mRNA levels that involved in the synthesis of fucosylated glycans.

FUT8 was strongly correlated with the presence of HCC tissues and HCC cells, and thus we speculated that FUT8 was a key factor in promoting malignant progression of HCC. In order to better understand the links between FUT8 and HCC progression, we further regulated FUT8 expression. FUT8 product decreased remarkably in MHCC97H shFUT8 cells, but increased in MHCC97L FUT8 cells labeled with FITC-LCA lectin. Furthermore, altered levels of FUT8 were shown to be involved in the proliferation, migration and invasion of MHCC97H and MHCC97L cells *in vitro*. Our results suggested that up-regulation of FUT8 was HCC progression-related. Altered FUT8 expression has impact on the remodeling of cell surface glycoproteins oligosaccharides, which may consequently affect the biological functions of tumor cells. Other findings demonstrated FUT8 were associated with advanced tumoral stage of HCC. Therefore FUT8 was implicated as a prognostic marker and therapeutic target for HCC [35, 37].

It is now recognized that the aberrant expression of various microRNAs is closely related to the clinical outcomes of several human cancers, including HCC. MiR-34a and miR-26a have been reported as one of the multicentric HCC-related miRNAs [21, 22, 23, 24]. Differentially expressed miR-455-3p has been evaluated in basal cell carcinoma (BCC) of the skin [38]. In this study, miR-34a, miR-26a and miR-455-3p were down-regulated in human HCC tissues compared with in adjacent tissues. Accordingly we also discovered that the expression of these miRNAs was reduced in MHCC97H cells compared with MHCC97L cells. Further experiments demonstrated that the regulated levels of miR-34a, miR-26a and miR-455-3p were demonstrated to be correlated with HCC cells progression both *in vitro* and vivo. Our data confirmed that miR-34a, miR-26a and miR-455-3p might act as tumor suppressors through regulating HCC cell progression.

Recent literature have shown that miRNAs as important regulators of glycosylation [39] can be used as a proxy to define the biological functions of glycosylation enzymes [40]. Vaiana *et al.* showed that MGAT4A (*N*acetylglucosaminyltransferase) was significantly altered in response to miR-424 in breast cell lines [41]. Moreover GalNAc transferase, GalNT7 was a target for miR-30 family, and ectopic expression of miR-30b/30d modulated the metastatic behavior of melanoma cells by directly targeting its enzyme activity [42]. In this study, our data confirmed the negative correlation between miR-34a, miR-26a and miR-455-3p downregulation and FUT8 upregulation. FUT8 has been validated as a direct target of miR-34a, miR-26a and miR-455-3p, in HCC tissues and HCC cell lines. These results corresponded to those results from Bernardi et al. who reported that ectopic expression of miR-34a was able to significantly decrease FUT8 levels and miRNAs were involved in the regulation of fucosylation machinery in HCC [43]. Interestingly, we also revealed that low expression of miR-34a, miR-26a and miR-455-3p, and high expression FUT8 were significantly associated with aggressive progression of human HCC cells. Functionally, these miRNAs were found to be involved in the development and progression of HCC through suppressing the expression of FUT8. These results not only verify the suppression effect of these miRNAs, but also suggest that the miRNAs combined with FUT8 might have a therapeutic potential for HCC treatment.

In conclusion, the current study showed that the *N*-glycan profiles and elevated fucosylation on the HCC tissues. The FUT family was found significantly different in transitional and tumor tissues, and two HCC cell lines with distinct metastatic potential. FUT8 was regarded as a potential target for HCC progression. The underlying mechanism was unraveled that the interaction between FUT8 and miR-34a, miR-26a and miR-455-3p led to fucosylation downregulation and subsequently HCC progression inhibition. Therefore FUT8/miRNAs pathway might be an ideal target for therapeutic intervention in HCC patients.

## MATERIALS AND METHODS

### Patients and tissue samples

The study and its informed consent have been examined and certified by the Ethics Committee of the First Affiliated Hospital of Dalian Medical University. Before collecting tumor specimens written informed consent was acquired from each enrolled patient. All specimens were handled anonymously according to the ethical and legal regulations.

Human primary HCC and adjacent tissues (3 cm from the tumor edge) were extracted from the same 27 patients who underwent surgical resections from June 2013 to April 2015 at the First Affiliated Hospital of Dalian Medical University (Dalian, China). The patients consisted of 19 men and 8 women, with age ranging from 19 to 78 years (mean age of 51.3 years). None of the patients received any chemotherapy or radiation treatment prior to the surgery. All samples were confirmed with pathological diagnosis and classified according to the 2012 hepatocellular carcinomas staging system of the International Union against Cancer (UICC). All samples were snap-frozen and stored in liquid nitrogen after collection. The clinicopathological factors of HCC are summarized in Table 2.

**Table 2:** Clinicopathological characteristics of HCC patients

Characteristics	*n*
**Group**	
Cancer tissues	27
Transitional tissues	27
**Gender**	
Male	19
Female	8
**Age (years)**	
≥ 50	17
< 50	10
**HBV infection**	
Negative	6
Positive	21
HCV infection	
Negative	25
Positive	2
**Cirrhosis**	
No	13
Yes	14
Serum AFP level (μg/L)	
≥ 200	18
< 200	9
Distant metastasis	
No	27
**Lymph node metastasis**	
Absent	27
**Clinical stage**	
I~II	27

### Preparation of N-glycans

Human primary HCC or adjacent tissues of 27 patients were assigned randomly into three groups, respectively (*n* = 9). The samples of per group were pooled. Membrane proteins were extracted from the three groups of tumor sample or three groups of adjacent tissue suspension using a CelLytic MEM Protein Extraction kit (Sigma, St Louis, MO, USA). The membrane protein concentration was measured with a Micro BCA Protein Assay kit (PIERCE, Rockford, IL). For releasing of N-glycans, 100 μg aliquots of lyophilized cell membrane proteins were first digested with trypsin (10 μg) and chymotrypsin (10 μg) dissolved in 25 mM ammonium bicarbonate (25 μL) at 37°C for 18 h. The digest was left in a water bath (85°C, 5 min) and after cooling N-linked oligosaccharides were released from peptides by treatment with PNGase F enzyme (2 μL; 6 U) at 37°C for 18 h followed by Pronase digestion (10 μg) at 37°C for 8 h. During the incubation time, the reaction sample was mixed occasionally. The released N-glycans were purified using an Oasis HLB cartridge (60 mg/3ml; Waters) and then were lyophilized. Permethylation was performed by using the solid NaOH technique.

### MALDI-TOF-MS analysis of permethylated N-glycans

For MS analysis, the dried permethylated sample was resuspended in 10 μL of acetonitrile. A total of 0.5 μL of matrix solution (10 mg of 2, 5-DHB dissolved in 1 mL of 30% ethanol) and 0.5 μL of the diluted analyte solution were spotted on the MALDI target plate (Bruker Daltonics). Then the plate was analyzed by MS, whose spectra were obtained from Na+ adduct ions. MALDI-TOF-MS spectra were acquired using an UltrafleXtreme^™^ mass spectrometer in the positive-ion reflector mode, controlled by FlexControl 3.4 software Build 119 (Bruker Daltonics). Monosaccharide compositions were determined by blasting against database GlycoMod: http://www.expasy.ch/tools/glycomod/.

### Cell culturation and transfection

Human hepatocarcinoma cell lines MHCC97H, MHCC97L and human normal liver cell line L02 were purchased from the KeyGEN Company (Nanjing, China). MHCC97H and MHCC97L cell clones of the same genetic background but with different metastatic potential. The three cell lines were grown in 90% Dulbecco Modified Eagle's Medium (DMEM, Gibco) supplemented with antibiotics (1× penicillin/streptomycin 100 U/ml, Gibco) and 10% heat-inactivated fetal bovine serum (FBS, Gibco). The cells were incubated in a humidified atmosphere of 5% CO_2_ at 37°C.

shRNA against FUT8, scrambled shRNA, miRNA-34a/miR-26a/miR-455-3p/ normal control (NC) mimics, and miRNA-34a/miR-26a/miR-455-3p/NC inhibitors were chemically synthesized by Shanghai GenePharmaCo., Ltd. (Shanghai, China). MHCC97H and MHCC97L cells were transfected with miRNAs (100 nM, the cell transfection efficiency was 72.3% ~78.5%) or shRNAs (50 nM, the cell transfection efficiency was 76.1%) using Lipofectamine 2000 Transfection Reagent (Invitrogen).

### RNA extraction and quantitative real-time PCR analysis

Total RNA was isolated from frozen tissues and HCC cell lines, using the RNeasy Mini Kit (QIAGEN, valencia, CA), and cDNA was synthesized using QuantiTect Reverse Transcription Kit (QIAGEN, valencia, CA) according to the manufacturer's protocol. The expression of miRNAs was determined by using mirVanaTM qRT-PCR microRNA Detection Kit (Ambion Inc., Austin, TX, USA) and normalized using the 2-^ΔΔCT^ method relative to U6-small nuclear RNA. FUT mRNAs were quantified with SYBR-Green-quantitative real-time PCR Master Mix kit (Toyobo Co., Osaka, Japan) and normalized to GAPDH, respectively. The expression level of target genes was determined by using Biosystems 7300 Real-Time PCR system (ABI, Foster City, CA, USA) and calculated as 2^−(Ct^_Target gene_^− Ct^_GAPDH_^)^. All assays were triplicated independently. The sequences of primers were as shown Table 3.

**Table 3:** qRT-PCR conditions and primer sequences for analysis of gene expression

Gene	Primer	Amplicon
***FUT1***	5′-AAAGCGGACTGTGGATCT-3′; 5′-GGACACAGGATCGACAGG-3′	168 bp
***FUT2***	5′-CTGCCCAACCACTCTGTC-3′; 5′-CCGTAAAGACAAAGAGGATG-3′	117 bp
***FUT3***	5′-CAACAGAGAAAGCAGGCA-3′; 5′-AAGAAACACACAGCCACC-3′	191 bp
***FUT4***	5′-TCCTACGGAGAGGCTCAG-3′; 5′-TCCTCGTAGTCCAACACG-3′	134 bp
***FUT5***	5′-ATGGCAGTGGAACCTGTC-3′; 5′-GCACCATCTCTGAGCAGC-3′	148 bp
***FUT6***	5′-CATTTCTGCTGCCTCAGG-3′; 5′-GGGCAAGTCAGGCAACTC-3′	138 bp
***FUT7***	5′-CCACGATCACCATCCTTG-3′; 5′-AGGCTTCGGTTGGCACTC-3′	118 bp
***FUT8***	5′-TCTAGCCGAGAACTGTCC-3′; 5′-GCTGCTCTTCTAAAACGC-3′	154 bp
***FUT9***	5′-AAATCCCATGCAGTTCTG-3′; 5′-AAACAAGTGCTCAATGCC-3′	124 bp
***FUT10***	5′-ATCTTGCCTGTGCGTCAC-3′; 5′-ATGCGTAGGTGCTTCCTC-3′	142 bp
***FUT11***	5′-CTCTTGGCTTTCTTGTCC-3′; 5′-ATGACGGAGTGATTGTTC-3′	167 bp
***POFUT1***	5′-AGATTCATGCCCACCTTGT-3′; 5′-GCTGTAGCCCACACACTGC-3′	140 bp
***POFUT2***	5′-TTCACGACCACTATGGAGG-3′; 5′-CGGAGCCCAGCTTGACCTT-3′	171 bp
***GAPDH***	5′-CTCCTCCACCTTTGACGCTG-3′; 5′-TCCTCTTGTGCTCTTGCTGG-3′	175 bp

### Western blot analysis

20 μg for each sample were run on a 10% SDS-PAGE and then transferred a polyvinylidene difluoride membrane (Pall Corporation). The membrane was blocked with 5% non fat dry milk in PBS containing 0.1% Tween 20 (PBST) for one hour and then probed with anti-FUT8 monoclonal antibody (Abcam, Cambridge, UK, 1:1000 dilution), or anti-GAPDH rabbit polyclonal antibody (Santa Cruz Biotech, Santa Cruz, CA, 1:1000 dilution). Detection was achieved using a secondary anti-rabbit HRP-conjugated IgG (Santa Cruz Biotech, Santa Cruz, CA, 1:1000 dilution). GAPDH was used as a control. Immunoreactive bands were visualised using ECL Western blotting kit (Amersham Biosciences, UK) and were normalized to those of GAPDH.

### Flow cytometry analysis

Cells were collected and washed thrice with PBS, and then centrifuged at 1000 r/min for 5 min in a 1.0 mL eppendorf tube. The cells were blocked in 2% BSA in PBS for 30 minutes and washed two times with PBS. After incubation of cells with fluorescein isothiocyanate (FITC)-LCA at a final concentration (10 μg/ml) in the dark for 40 min at room temperature, residual unbound FITC-LCA was then discarded by repeat centrifugation of samples at 1000 r/min. After removal of supernatant, cells were resuspended in 0.2 ml PBS. The control, which was negative, cells and FITC-LCA was alone. Cells were collected and analyzed with Flow Cytometer (BD FACSAria, San Diego, CA, USA). Experiments were repeated at least 3 times with similar results each time.

### Cell counting kit-8 (CCK-8) assays

The cell proliferation assays were performed using cell counting kit-8 (CCK-8; KeyGEN, Nanjing, China) according to the manufacturer's instruction. Cells (1 × 10^3^/well) were seeded in 96-well plates with 100 μl of DMEM medium containing 10% FBS and cultured in a humidified incubator (at 37°C, 5% CO_2_) for 24, 48 and 72 hrs, Then, each well was added 10 μl CCK-8 solutions at 37°C for 2 hrs. The absorbance at 450 nm was immediately measured using a microplate reader. Each experiment was performed at least 3 times.

### Focus formation assay

Effect of miRNA mimic or inhibitor on foci formation abilities of the HCC cells was assessed by focus formation assays. The assay was applied in 6-well plates. Cells (1 × 10^3^) were trypsinized to single-cell suspension and placed in triplicate onto plastic culture dishes in DMEM containing 10% FBS. The cultures were maintained in the same medium, with medium changes every 3 days, until the appearance of foci from transformed cells was evident (7 days after transfection). Then the colonies were counted with crystal violet staining.

### Immunofluorescence analysis

Cells were transfected with miRNA mimic or miRNA inhibitor as described in above. Cells were fixed with cold 4% formaldehyde for 10 min at room temperature and subsequently washed three times with PBS. Then, the cells were permeabilized with PBS containing 0.3% triton X-100 and 2% BSA for 30 minutes at room temperature. The cells were incubated with primary antibody against Ki67 (Abcam, Cambridge, MA, USA) overnight at 4°C. After washing with PBS, cells were incubated with secondary antibody. The cells were washed with PBS and incubated with 1 μg/mL of 4, 6-diamino-2-phenylindole (DAPI, Sigma-Aldrich, St Louis, MO, USA) for nuclear staining. Images were generated on a fluorescence microscope (OLYPAS).

### Cell invasion and migration assays

The invasion abilities of human HCC cells transfected with FUT8 shRNA/control shRNA, miR-34a/miR-26a/miR-455-3p/NC mimic or miR-34a/miR-26a/ miR-455-3p/NC inhibitor were tested by invasion assays, respectively, using 24-well transwell units (Corning, NY, USA) with 8μm pore size polycarbonate filter coated with ECMatrix gel (Chemicon) to form a continuous thin layer. Cells (4 × 10^4^) were harvested in serum-free DMEM and added to the upper chamber. The lower chamber contained 500 μl DMEM with 10% (vol/vol) FBS. The cells were incubated at 37°C, 5% CO_2_ incubator for 24 h. At the end of incubation, the invaded cells at the reverse side of the insert were fixed in methanol and were stained with Wright-Giemsa. The number of invaded cells on the lower side of the membrane was counted at 400× magnification from ten different fields of each filter. The migration assay was conducted following the aforementioned steps, except for the absence of the Matrigel, and 4 × 10^4^ cells were added to the upper chamber. Each experiment was performed in triplicate and repeated 3 times.

### Tumor xenograft models

Five-week-old female athymic nude mice were obtained from Animal Facility of Dalian Medical University, and used for subcutaneous tumor implantation. Approximately 1 × 10^7^ cells were inoculated subcutaneously into the right flank of each nude mouse, respectively. One week later, the mice were injected intratumorally with miR-26a/miR-34a/miR-455a mimics or mimic control three times per week for 3 weeks respectively. Measurements of tumor size began in the first week of postinoculation and monitored weekly by measuring the perpendicular tumor diameters, length (L) and width (W), with a vernier caliper. Mice were killed under anesthesia 4 week after injection. Mice were sacrificed and their tumors were isolated, photographed and weighed. Tumor size was measured using calipers and recorded following the formula: (length × width^2^)/2.

### Immunohistochemical (IHC) analysis

After the xenograft tumor being harvested, it was immediately fixed in 4% paraformaldehyde, dehydrated in a graded series of alcohol, and then embedded in paraffin. 5 μm sections were sliced, dried, deparaffinized, rehydrated and then were immersed in 3% hydrogen peroxide for 10 min to block endogenous peroxidase. After consecutive washing with PBS, the slices were incubated with primary anti FUT8 or Ki67 antibody (1:200, Abcam, Cambridge, UK) at 4°C overnight. The secondary streptavidin-HRP-conjugated antibody staining (Santa Cruz Biotech, Santa Cruz, CA) was performed at room temperature for 60 min. Finally, the sections were counterstained with hematoxylin and cover-slipped. The Image-ProPlus 4.5 Software (Media Cybernetics, USA) was used to analyze the expression of proteins.

### Luciferase assays

A pmirGLO Dual-Luciferase miRNA Target Expression Vector was chosen for 3′UTR Luciferase assays (Promega, Madison, WI, USA). The vector contained firefly luciferase (luc2) used as primary reporter to monitor mRNA regulation and Renillaluciferase (hRlucneo) acting as a control reporter for normalization and selection. The vector could be used to study the influence of miRNAs on transcript stability and activity by the insertion of miRNA target sites 3′ untranslated region (UTR) of gene. The wild-type FUT8 and mutant FUT8 3′-UTR were specifically synthesized (Promega) and inserted into the vector. HEK 293T cells of 50% confluence were seeded (5 × 10^4^ cells per well) in a 24 well dish and were transfected using Lipofectamine 2000. The miRNA mimic or NC mimic with pmirGLO-FUT8 3′-UTR wt vector, pmirGLO-FUT8 3′-UTR mut vector or empty vector were co-transfected per well. Luciferase assays were performed up to 48 h after transfection by using the dual luciferase reporter assay system (Promega) according to the manufacturer's protocol. Firefly and Renilla luciferase activities were measured and normalized to Renilla luciferase. The mean of relative luciferase activities from the cells transfected with the empty vector and NC mimic was set at 100. The results were presented as the mean value ± SD for three repeat experiments.

### Statistical analysis

Each experiment was performed at least in triplicate, and the measurements were performed in three independent experiments. Data are expressed as means ± standard deviation (SD). Student's *t*-test was used to compare the means of two groups. *P* < 0.05 was considered statistically significant. All analyses were performed using SPSS 17.0 statistical packages (SPSS Inc., Chicago, IL).
